The article "A Pneumonia Diagnosis Scheme Based on Hybrid Features Extracted from Chest Radiographs Using an Ensemble Learning Algorithm" was published in 2021. Journal: J Healthc Eng.

# A Pneumonia Diagnosis Scheme Based on Hybrid Features Extracted from Chest Radiographs Using an Ensemble Learning Algorithm

**DOI:** 10.1155/2021/8862089

**Published:** 2021-02-25

**Authors:** Mehedi Masud, Anupam Kumar Bairagi, Abdullah-Al Nahid, Niloy Sikder, Saeed Rubaiee, Anas Ahmed, Divya Anand

**Affiliations:** ^1^Department of Computer Science, College of Computers and Information Technology, Taif University, P.O. Box 11099, Taif 21944, Saudi Arabia; ^2^Computer Science and Engineering Discipline, Khulna University, Khulna 9208, Bangladesh; ^3^Electronics and Communication Engineering Discipline, Khulna University, Khulna 9208, Bangladesh; ^4^Department of Industrial and Systems Engineering, University of Jeddah, P.O. Box: 80327, Jeddah 21589, Saudi Arabia; ^5^Department of Computer Science and Engineering, Lovely Professional University, Punjab 144411, India

## Abstract

Pneumonia is a fatal disease responsible for almost one in five child deaths worldwide. Many developing countries have high mortality rates due to pneumonia because of the unavailability of proper and timely diagnostic measures. Using machine learning-based diagnosis methods can help to detect the disease early and in less time and cost. In this study, we proposed a novel method to determine the presence of pneumonia and identify its type (bacterial or viral) through analyzing chest radiographs. We performed a three-class classification based on features containing diverse information of the samples. After using an augmentation technique to balance the dataset's sample sizes, we extracted the chest X-ray images' statistical features, as well as global features by employing a deep learning architecture. We then combined both sets of features and performed the final classification using the RandomForest classifier. A feature selection method was also incorporated to identify the features with the highest relevance. We tested the proposed method on a widely used (but relabeled) chest radiograph dataset to evaluate its performance. The proposed model can classify the dataset's samples with an 86.30% classification accuracy and 86.03% F-score, which assert the model's efficacy and reliability. However, results show that the classifier struggles while distinguishing between viral and bacterial pneumonia samples. Implementing this method will provide a fast and automatic way to detect pneumonia in a patient and identify its type.

## 1. Introduction

Pneumonia refers to severe inflammation caused by infections inside the lungs, which are crucial organs of the respiratory system. These infections can be caused by several infectious agents, including bacteria, viruses, and fungi, and can occur in one or both lungs. These infections fill the minuscule air-sacs inside the lungs (called alveoli) with fluid and pus, restricting them to get oxygen-rich air that we breathe in. As a result, breathing for the patient becomes increasingly difficult and painful. A pneumonia patient may also experience other symptoms such as fever, dry cough, vomiting, exhaustion, and chest pain [1]. The effects of pneumonia can range from mild infections to lethal organ failure, depending on the severity of the condition, the patient's age, and his/her immune system. Apart from infants and toddlers, people with asthma, diabetes, chronic obstructive pulmonary disease (COPD), sickle cell disease, the history of other heart-related problems, and smoking habit have a higher chance of getting pneumonia.

The article "A Pneumonia Diagnosis Scheme Based on Hybrid Features Extracted from Chest Radiographs Using an Ensemble Learning Algorithm" was published in 2021. Journal: J Healthc Eng.

Every year pneumonia kills more than two million people worldwide, most of whom are children under five years of age and people over 70 [2]. However, studies found that half the deaths from a particular bacterial pneumonia occur in people between 18 and 64 years in the USA [3]. The rate of death due to pneumonia is highest in the countries of sub-Saharan Africa and the Southeast Asia region. The economy of a country has a clear link with its pneumonia mortality rate [4]. The mortality rate is as high as one in 100 people in some developing countries, compared with one in 1000 people in the developed ones. In 2017, more than half of child deaths due to pneumonia occurred in only five countries—India, Pakistan, Nigeria, Ethiopia, and the Democratic Republic of Congo—all of which have the majority of their population living below the poverty line [2]. In 2018, Watkins and Sridhar called pneumonia the ultimate disease of poverty [4]. Malnutrition, poor and dense living conditions, air pollution, and untreated heart conditions are reasons for such high pneumonia mortality rates in countries with low incomes.

Several bacteria, viruses, and fungi can cause pneumonia, among whom the bacterium *Streptococcus pneumoniae* is responsible for most cases. Pneumonia is a contagious disease that often affects multiple community members through the spread of its germs. The diagnosis of pneumonia is mostly made based on the associated symptoms and some physical examination. Among the effective and proven diagnostic methods, chest X-rays, sputum culture, and blood tests are most common. The treatment of pneumonia relies on several factors, such as the patient's age, the extent and duration of the infection, and the type of pneumonia (i.e., viral pneumonia, bacterial pneumonia, or others). Since the disease is easily spreadable and the associated symptoms are not always apparent or severe, patients with pneumonia often go undiagnosed. The rate of undiagnosed cases is particularly high in developing countries as the poor often cannot afford to pay for the diagnosis. Moreover, many regions of these countries lack the proper equipment, facilities, or qualified individuals required to carry out the diagnosis. These factors increase the chance of the disease advancing towards the severe stages and, consequently, decrease the patients' chances of survival.

The article "A Pneumonia Diagnosis Scheme Based on Hybrid Features Extracted from Chest Radiographs Using an Ensemble Learning Algorithm" was published in 2021. Journal: J Healthc Eng.

The emergence of powerful machine learning and artificial intelligence techniques has provided an alternative way to diagnose pneumonia using computers. Machine learning-based diagnostic methods are fast, automatic, cost-efficient, and suitable for rapid utilization. Although the use of computers in disease diagnosis dates back to the 1960s, the area is currently far more promising because of the advancements in computer technology and the development of new and capable machine intelligence algorithms [1]. Especially, convolutional neural network- (CNN-) based deep learning algorithms have shown astounding success while working with high-dimensional data such as medical images and videos. Multimodality image fusion techniques have improved these medical imaging methods' efficacy by allowing us to obtain more informative image samples [5]. Researchers have been testing and reporting CNN-based pneumonia diagnosis methods for over a decade, and some of the recent ones are truly promising. However, most of these methods only deal with the challenge of determining pneumonia, not identifying its type, which can be inconvenient as the treatment procedure depends on it. Identifying the cause of pneumonia at an early stage will help the physicians to devise more effective treatment plans for their patients and increase their chances of recovery.

To tackle this issue and provide an alternative means of pneumonia diagnosis, this study describes a novel machine learning-based method for detecting pneumonia and its type using the RandomForest classifier, a popular supervised learning algorithm capable of delivering excellent classification outcomes. Manual and automatic features were extracted from chest X-ray images using a statistical and deep learning method to provide the classifier with distinctive and manifold information on the samples. We tested the proposed method on a subset of a benchmark chest radiograph dataset widely used for pneumonia detection. The acquired results show that the proposed model can carry out the intended classification with acceptable accuracy and a reasonable degree of reliability. Integrating this method with the concurrent diagnostic measures will allow medical professionals to automate the initial diagnosis and have a second opinion, which might help provide treatments to a larger group of patients.

The article "A Pneumonia Diagnosis Scheme Based on Hybrid Features Extracted from Chest Radiographs Using an Ensemble Learning Algorithm" was published in 2021. Journal: J Healthc Eng.

The rest of the study is organized as follows.  Section 2 describes the dataset employed in this study and a few recent works in pneumonia diagnosis along with their outcomes.  Section 3 outlines the methodology of the proposed automatic diagnosis method and discusses its building blocks.  Section 4 presents the acquired result of the proposed method with necessary discussion, judges the outcomes based on some widely used evaluation metrics, and compares its performance with other contemporary methods. Finally, Section 5 highlights the contributions of the study and lists some possible future works.

## 2. Employed Dataset and Prior Works

This study used a chest radiograph image dataset collected from a Kaggle repository entitled “Chest X-rays: bacterial/viral pneumonia/normal,” which was published in October 2020 [6]. The dataset contains 4672 labeled samples (for training) divided into three classes—no disease, bacterial pneumonia, and viral pneumonia. The dataset is a relabeled version of the popular dataset entitled “Chest X-ray Images (Pneumonia),” which contains 5863 labeled images [7]. However, samples of the latter dataset are categorized into two classes—normal (N) and pneumonia (P). To construct this dataset, a total of 5232 chest radiographs were collected from infected and healthy children; 3883 of them were characterized as depicting pneumonia [8]. As the pneumonia-positive samples also contain information on whether it is bacterial or viral, the authors further divided the class samples into bacterial pneumonia and viral pneumonia, making it a three-class classification problem. However, in the relabeled version, they put 20% of the original samples into the testing subset (for the competition) without providing their associated labels.  Figure 1 shows a few samples of the dataset that belong to three different classes.

The original dataset was published in 2018, and since then, about 100 research articles have been published so far involving its samples [9]. The baseline study by Kermany et al. reports a classification accuracy of 92.8% using the Inception V3 architecture (pretrained on the ImageNet dataset) while distinguishing between normal and pneumonia samples [8]. They had an accuracy of 90.9% while distinguishing between bacterial and viral pneumonia. However, recent studies have reported better classification outcomes (for binary classifications) on this dataset. For example, in 2020, Chouhan et al. reported a study describing a transfer learning-based approach for pneumonia detection, which resulted in a 96.39% classification accuracy [10]. They used five different pretrained CNN architectures for feature extraction and an ensemble technique for the final classification. Mittal et al. used dynamic capsule routing to achieve a maximum classification accuracy of 95.90% using the original dataset [11]. Nahid et al. proposed a pneumonia detection method employing a two-channel CNN, which achieved a classification accuracy of 97.92% [1]. The authors used multiple image processing techniques to process the samples before performing the classification using the deep learning model. Siddiqi presented PneumoniaNet—a CNN-based architecture with 21 layers including normal and depthwise separable convolution operations [12]. Multiple binary classifications were performed in that study to detect pneumonia, and PneumoniaNet achieved a 94.80% classification accuracy on the testing samples. Hu et al. proposed a multikernel depthwise convolution scheme named MD-Conv for pneumonia detection [13]. They tested their method on the popular Chest X-ray 14 dataset and achieved a 98.30% area under the curve (AUC) score. In 2019, Stephen et al. presented a binary classification scheme to classify the samples of the chest X-ray images (pneumonia) dataset using a customized deep learning architecture with four 2D-convolutional and four 2D-MaxPooling layers [14]. They achieved the best classification accuracy (93.73%) when the input images of the model had a shape of 200 × 200 × 3.

The article "A Pneumonia Diagnosis Scheme Based on Hybrid Features Extracted from Chest Radiographs Using an Ensemble Learning Algorithm" was published in 2021. Journal: J Healthc Eng.

A few studies performed three-class classification using chest X-ray images, similar to the proposed approach, involving the original dataset. For instance, in 2020, Mahmud et al. described CovXNet (multidilation CNN) for pneumonia and COVID-19 detection and pneumonia classification [15]. They performed multiple classifications using various subsets of two chest radiograph datasets and using multiple deep learning architectures. However, they achieved peak results by using CovXNet with transferable multireceptive feature optimization. Jain et al. performed three-class classifications to identify pneumonia and its types using CNN and transfer learning [16]. Like the previous study, they experimented with six different CNN-based models to achieve their task, among which four were pretrained models.

In recent studies, many researchers are combining this dataset's images with other COVID-19 cases to determine whether the patient has typical pneumonia or COVID-19. For example, in 2021, Karakanis and Leontidis described two deep learning models with a lightweight architecture to detect COVID-19 and bacterial pneumonia [17]. Their research overcame the scarcity of COVID-19 samples by generating synthetic chest X-ray images using a conditional generative adversarial network (cGAN). In 2020, Khalifa et al. presented a study based on neutrosophic set significance learning models on deep transfer learning. They experimented with the samples of the described dataset along with another COVID-19 dataset [18]. Their study focused on observing the effect of varying the train-test ratio on the classification performance while using three popular deep transfer learning models: AlexNet, GoogLeNet, and ResNet18. They achieved peak performance (87.10% classification accuracy) when they used 90% of the available samples to train AlexNet on indeterminacy domain images. Apart from the chest X-ray images (pneumonia) dataset, other chest X-ray datasets are also being used for pneumonia and COVID-19 diagnosis. For instance, in 2020, Singh et al. used deep CNNs to classify the samples of two COVID-19 datasets with the aim to identify the disease based on the information present in their corresponding chest radiographs [19]. And Gianchandani et al. described two ensemble deep transfer learning-based pretrained models for pneumonia and COVID-19 diagnosis [20]. In their study, they ensembled the outputs of modified VGG16 and ResNet152V2 architectures for COVID-19 detection and the outcomes of modified VGG16 and DenseNet201 architectures for the separation of healthy, pneumonia, and COVID-19 samples.

The article "A Pneumonia Diagnosis Scheme Based on Hybrid Features Extracted from Chest Radiographs Using an Ensemble Learning Algorithm" was published in 2021. Journal: J Healthc Eng.

## 3. Methodology

The employed methodology involves several steps. First of all, an image augmentation operation was performed on two classes' samples to balance the dataset. Then, the chest X-ray images were resized to make them uniform in terms of their resolution. After that, features were extracted from them using a statistical and a deep learning technique. Upon extraction, these sets of features were concatenated to construct the final set of features. Finally, based on these features, the samples were categorized using the RandomForest classifier. Furthermore, a genetic algorithm was used for feature selection to reduce the dimension of data. Another classification was performed based on these selected features to point out how much the omission of features has affected the model's performance.  Figure 2 outlines the workflow of the described method. It has four main stages: data collection and preliminary processing, feature extraction, feature concatenation and selection, and samples classification with performance evaluation. The first step involves a simple image augmentation technique. The second step involves two image processing—image histogram and two-dimensional discrete wavelet transform (2D DWT)—and a deep learning algorithm. The third step involves a genetic algorithm for feature selection. And the last step involves the RandomForest classifier as the ultimate learning algorithm.

The article "A Pneumonia Diagnosis Scheme Based on Hybrid Features Extracted from Chest Radiographs Using an Ensemble Learning Algorithm" was published in 2021. Journal: J Healthc Eng.

### 3.1. Balancing Out the Sample Sizes

Table 1 shows the number (and percentage) of samples of each class present in the original dataset. It also declares the labels we assigned to classes to refer to them afterward. As we can see, the dataset is highly imbalanced since Class B has almost twice the sample size of the other two. Carrying out classification at the present state can make the classifier's decision biased towards the majority class. Qu et al. assessed the effects of class imbalance and how to mitigate them using two chest X-ray datasets [21]. We augmented the samples of the two minor classes (classes H and V) by 180° and added the resultant images to the original ones to mitigate this issue. As the table shows, it mostly solved the class imbalance problem. We also resized all the images to 256 pixels × 256 pixels (in width and height).

### 3.2. Statistical Feature Extraction

As mentioned earlier, we calculated the histogram of the chest radiographs and used that information as the statistical features that represent their corresponding samples. The histogram simply yields at what frequency each gray level occurs within a grayscale image. Since we are working with 8 bit images, their intensity values range from 0 (black) to 255 (white). If we consider *g*_*i*_ as the *i*^th^ gray level and *n*_*i*_ as the number of pixels with that particular gray level, the probability density of *g*_*i*_ can be defined as follows:

(1) $$\begin{array}{c} P\left(g_{i}\right)=\frac{n_{i}}{256\times 256}, \end{array}$$

since we are working with 256 pixel × 256 pixel images [22]. The graphical appearance of equation (1) is called the histogram of the image. Its cumulative distribution function is defined as follows:

(2) $$\begin{array}{c} C\left(g_{i}\right)=\sum_{0}^{255}P\left(g_{i}\right). \end{array}$$

### 3.3. Deep Feature Extraction

We extracted convolutional features from the image samples to capture the information that a deep learning model would use to learn their underlying properties. Prior to that, we performed a domain transformation operation on the X-ray images. We transformed these chest images using the 2D DWT to reveal the frequency and spatial properties of that image at the same time. The 2D DWT algorithm decomposes an image using a high-pass filter and a low-pass filter into four coefficients: the approximate coefficients, the horizontal vertical detail coefficients, and the diagonal detail coefficients. The approximate coefficients of a level can be further processed to achieve higher-level decompositions. Among the four coefficients, the approximate coefficients contain the most amount of information on the input images. In this study, we used these coefficients of the chest radiographs for information. For a sample image *I*, its approximate coefficients can be calculated using

(3) $$\begin{array}{c} cA_{i+1,\left(x,y\right)}=\frac{1}{2}\sum_{k=0}^{255}\sum_{l=0}^{255}d_{k}d_{l}cA_{i,\left(2x+k,2y+l\right)}, \end{array}$$

where *b* and *d* are the scaling coefficients, *k* and *l* are the scaling-coefficient indices, *x* and *y* are the location indices, and *i* is the decomposition level [23]. Each level of decomposition reduces the size of the original image to its half. Hence, this domain transformation provided us samples having a dimension of 128 pixel × 128 pixel. We then passed these images to a deep learning model to extract features from them.  Figure 3 outlines the architecture of the deep learning model we designed to extract deep features. It incorporates four two-dimensional convolutional layers (Conv2D), four two-dimensional MaxPooling layers (Max_pooling2D), three dropout layers, and two batch normalization layers. It also shows the shape of a sample image as it passes through each layer.

The article "A Pneumonia Diagnosis Scheme Based on Hybrid Features Extracted from Chest Radiographs Using an Ensemble Learning Algorithm" was published in 2021. Journal: J Healthc Eng.

In the convolution layer, numerous kernels are derived and then compared to different parts of an image. A convolution operation, (*x*^*∗*^*ω*)(*a*), of functions *x* (called the input) and *ω* (called the kernel) can be defined as

(4) $$\begin{array}{c} \left(x{}^{*}\omega \right)\left(a\right)=\int x\left(t\right)\omega \left(a-t\right)\text{d}a, \end{array}$$

and for discrete convolution, assuming that *t* is discrete,

(5) $$\begin{array}{c} \left(x{}^{*}\omega \right)\left(a\right)=\sum_{a}x\left(t\right)\omega \left(t-a\right), \end{array}$$

where *a* ∈ **R**^*n*^ for all *n* ≥ 1, a higher-dimensional variant replaces the integral [24]. Now, in the case of two-dimensional images, we need to rewrite equation (5) as follows:

(6) $$\begin{array}{c} \left(I{}^{*}K\right)\left(i,j\right)=\sum_{p=0}^{m-1}\sum_{q=0}^{m-1}I\left(p,q\right)K\left(i-p,j-q\right), \end{array}$$

where *I* is a sample image with a resolution of *m* × *m* pixels. The output of a convolution layer is called a feature map. The job of a pooling layer is to reduce the size of the feature map without losing vital information. We used MaxPooling in our architecture. Given a block of the feature map, MaxPooling keeps only the maximum value of that block. If a MaxPooling operation is performed with a (*p* × *p*) kernel and *p* stride on a (*i* × *j*) feature map, it will result in a (*i*/*p* × *j*/*p*) feature map. Dropout and batch normalization help to reduce overfitting while training the model. At the final layer of the model, all the extracted features were flattened to get a vector of features, which was used to represent the samples later on.

The article "A Pneumonia Diagnosis Scheme Based on Hybrid Features Extracted from Chest Radiographs Using an Ensemble Learning Algorithm" was published in 2021. Journal: J Healthc Eng.

### 3.4. Feature Concatenation and Selection

We acquired 256 features from each image containing its gray level information and 576 features containing the aggregated information due to numerous convolutions on the image. In this step, we combined these two sets of features (832 in total) to make both types of information available to the learning algorithm.

All the features present in the combined dataset do not contain the same level of classifiable information and are not useful to the learning algorithm. That is why we attempted to identify the best set of features within the combined set we created earlier. We used an evolutionary algorithm named the genetic algorithm for feature selection. As the name suggests, the algorithm is inspired by the process of natural selection and borrows most of its jargon from biology. The flow chart of a typical genetic algorithm's operations is depicted in Figure 4. As the figure shows, the algorithm starts with a random population. The members of a population can spread throughout the search space. Three of its primary operations on the population are selection, crossover, and mutation [25]. The algorithm tries to converge towards the global optimum over a series of steps called generations. Selection makes sure that better performing or “fitter” members of the current population are propagated towards the next generation, whereas the weaker members are excluded, which strengthens the next generation. Crossover allows multiple individuals to exchange information creating new solutions, some of which might be better than the initial ones. Mutation randomly alters the genes of an individual to create new solutions. A new population is devised by performing these operations on the previous one. The process is repeated until a particular convergence criterion is met, a predefined number of generations are elapsed, or if the solution remains the same for a few consecutive generations.

### 3.5. Using RandomForest for Classification

Developed based on Breiman's idea of “Bagging,” RandomForest is a decision tree-based ensemble learning algorithm widely used to solve classification and regression problems [27]. It is comprised of numerous individual trees, each of which provides an independent class prediction. The algorithm then performs voting on the trees' decisions, and the winning class becomes the model's prediction. RandomForest improves its decision-making capacity by relying on the “wisdom of the crowds.” Let us consider a dataset *𝒮*={(*x*_*i*_, *y*_*i*_)}, where *x* represents a sample and *y* represents a feature. Also, the dataset has *𝒩* samples and ℳ features in each sample. Then, to classify the samples of the dataset, the RandomForest follows these steps [28]:

Step 1: *t* training subsets are created from the primary dataset (*𝒮*) following the principles of bootstrap sampling. Every time, randomly *𝒩* records are selected from *𝒮*. The resultant training set can be expressed as follows:
  (7) $$\begin{array}{c} S_{Tr}=\left\{S_{1},S_{2},\ldots .S_{t}\right\}. \end{array}$$
(i) Records that are not selected every time are put into another dataset, called the out-of-bag (OOB) dataset. Therefore, *t* OOB datasets are also generated in this step alongside *𝒮*_*Tr*_. These sets are used to test the model after learning.
  (8) $$\begin{array}{c} S_{\text{OOB}}=\left\{{\text{OOB}}_{1},{\text{OOB}}_{2},\ldots ,{\text{OOB}}_{t}\right\}, \end{array}$$
Here *t* ≪ *𝒩* and *𝒮*_*j*_ ∪ OOB_*j*_=*𝒮*.
Step 2: at this step, multiple decision trees are created following the C4.5 or CART algorithm from each *𝒮*_*i*_. While growing these trees, *m* features are randomly selected from ℳ. Splitting of the tree nodes depends on the gain of each feature. Splitting continues until the generation of a leaf node. *t* decision trees are similarly trained from *t* subsets.
Step 3: the decision of the *t* trees are collected and aggregated as follows:
  (9) $$\begin{array}{c} H\left(X,\Theta j\right)=\sum_{i=1}^{t}h_{i}\left(x,\Theta j\right), \end{array}$$
Where *j* ={1,  2,…, *m*}, and *X* denotes the set of input features. *H*(*X*, Θ*j*) is a metadecision tree classifier where Θ*j* determines the growth of the tree.

The article "A Pneumonia Diagnosis Scheme Based on Hybrid Features Extracted from Chest Radiographs Using an Ensemble Learning Algorithm" was published in 2021. Journal: J Healthc Eng.

## 4. Results and Discussion

In this study, we performed a three-class classification to determine the presence of pneumonia and its type. In this section, we present the acquired results of classification. As discussed earlier, we extracted two different sets of features from the available chest X-ray images. We performed multiple classification operations to highlight how using diverse sets of features has changed the classification outcome. To train our supervised learning algorithm, we assigned 70% samples of the dataset (4974 samples) to the training subset, based on which the learning model was built. Then, we tested the model's capacity on the remaining 2132 samples, which belonged to the testing subset. The selection of samples during the split was random, and the two subsets did not have any common samples.

First, the deep learning model illustrated in Figure 3 was trained based on the training subset to extract the convolutional features. Four dense layers were appended to the end of the architecture to perform classifications of the training samples. The model was trained for 100 epochs.  Figure 5 presents the corresponding loss values at each epoch in the training stage. As seen from the figure, the loss decreased gradually as the model was further trained, which indicates the improvement in the model's performance while classifying the samples of the training subset. After being trained for 100 epochs (minimum loss), the global features were extracted from the layer marked in Figure 3.

The article "A Pneumonia Diagnosis Scheme Based on Hybrid Features Extracted from Chest Radiographs Using an Ensemble Learning Algorithm" was published in 2021. Journal: J Healthc Eng.

### 4.1. Performance of the Proposed Method

Table 2 presents the outcomes of the classifications performed on the testing subset based on different sets of features. Before performing these classifications, the employed RandomForest classifier was mildly tuned to reduce overfitting while learning from the training samples. The values of the RandomForest's parameters that were tuned for optimal performance on the dataset are presented in Table 3. For each classification, the classifier was trained on the corresponding set of features. As seen from the table, the model performed the best when both sets of information (statistical and deep) were available to it. The combined set of features helped the model learn about the samples more thoroughly, allowing the model to classify the samples of the testing subset with more success. Numerically, the model was able to correctly identify 86.30% samples of the testing subset while both sets of features were used, which is 4.17% and 3.28% higher than when only the histogram and convolutional features were used, respectively.

Table 2 also provides the precision, sensitivity, specificity, and F-scores of the performed classifications. Since we are working with a slightly imbalanced dataset, these metrics are essential to comprehend the classifier's actual performance. The F-score, which is a weighted average of the precision and sensitivity scores, is not affected by the bias classifier faces because of the class imbalance; hence, it is often considered a better evaluation metric than the accuracy. As we can see, the F1-scores closely follow the accuracy scores and indicate that, indeed, the model's performance improved when the combined set of features was used. The values of these metrics also assure the acquired results' authenticity as well as the proposed model's reliability.

As mentioned in the previous section, we employed a genetic algorithm to reduce the number of features while sacrificing performance as minimally as possible. The algorithm allowed us to identify a set of 425 features of the highest importance among the extracted 832 features.  Figure 6 shows the fitness values of numerous populations considered by the genetic algorithm. We used the classification accuracy as the fitness function of the algorithm to evaluate each population. We set the algorithm to run for 50 generations, and as the figure indicates, among them, the 45^th^ generation was the fittest one. The feature set of that generation was collected for further operations. Table 2 also provides the classification outcomes based on this selected set of features. Compared with the performance based on the combined feature set, the feature omission yields a 0.51% and 0.52% decrease in accuracy and F-score, respectively. This trade-off is acceptable, considering that it allowed us to reduce 49% of the features in exchange for a marginal decline in the model's performance.

The article "A Pneumonia Diagnosis Scheme Based on Hybrid Features Extracted from Chest Radiographs Using an Ensemble Learning Algorithm" was published in 2021. Journal: J Healthc Eng.

Figures 7 and 8 present the confusion matrices and classwise receiver operating characteristics (ROC) curves, respectively, based on different sets of features used for classification. These measures can help us analyze the model's performance in-depth and identify the areas of success and failure of the described classifier. As seen from the Figures 7(c) and 7(d), most healthy samples were correctly identified by the classifier. However, the latter classes' samples (bacterial and viral pneumonia) confused the classifier the most. These phenomena are reflected in Figures 8(c) and 8(d) as well. They show that, in both cases, Class H had an AUC score of 98%, indicating a very high true-classification rate of the class. However, classes B and V have slightly lower AUC scores, meaning there is room for improvement, especially while classifying these classes' samples.

Table 4 presents the classification's individual classwise performance (based on the combined set of features) in terms of the parameters discussed above. As seen from the table, Class B suffers from low sensitivity compared to the other classes' scores. Apart from that, the precision and specificity scores are quite consistent. The poor sensitivity of Class B has affected its F-score as well. As discussed earlier, this is the area where the performance of the proposed method can be improved.

### 4.2. Performance Comparison

To put the model's performance into context, we have compared it with similar methods as shown in Table 5. The first six studies of the table [1, 8, 10–14] perform only binary classifications to determine the presence of pneumonia or its type. Hence, their reported results are not directly comparable to ours. References [15, 16] perform three-class classifications using multiple deep learning methods. Two of their reported models achieved higher accuracy scores than ours (91.70% and 92.31%), and at one instance, the performance of the described model was almost identical to our proposed method (86.30%). Our method outperforms the presented results in those studies in terms of classification accuracy in all the other cases. However, we want to mention that none of the cited studies deal with the exact dataset used in this study. In most cases, they took the associated class samples from the parent dataset.

The article "A Pneumonia Diagnosis Scheme Based on Hybrid Features Extracted from Chest Radiographs Using an Ensemble Learning Algorithm" was published in 2021. Journal: J Healthc Eng.

## 5. Conclusion

This study describes a novel pneumonia diagnosis method that focuses on the benefits of extracting diverse (statistical and convolutional) features from chest radiographs and combining them for classification, which was performed by an ensemble learning algorithm. The acquired results show that the classifier is capable of providing an 86.30% classification accuracy and 86.03% F-score while tested on a widely used (but recently relabeled to create an extraclass) dataset. The data dimension was reduced by employing a feature selection algorithm, which had a negligible effect on the method's performance. However, the performance can be further improved, especially while separating viral and bacterial pneumonia classes' samples. We look forward to exploring more statistical and deep features (with different deep learning architectures) and focusing on hypertuning the classification algorithm more sophisticatedly to overcome the shortcomings (of this method) in our future studies. Further research can also be conducted by combining the samples of this dataset with similar chest X-ray datasets (which may contain other classes) to increase the amount of training data to learn from, which will lead to better and more capable diagnosis methods. Practical implementation of the devised pneumonia diagnosis methods (while keeping real-world constraints in mind) to help the medical professionals will benefit the mass population, especially the children of the low-income countries.

## Figures and Tables

**Figure 1:** Sample images of class showing (a) no disease, (b) bacterial pneumonia, and (c) viral pneumonia.

**Figure 2:** Workflow of the proposed pneumonia identification method.

**Figure 3:** Architecture of the model used for deep feature extraction.

**Figure 4:** Workflow of the genetic algorithm [26].

**Figure 5:** The training loss curve.

**Figure 6:** Fitness values of the population of the genetic algorithm.

**Figure 7:** Confusion matrices of the classification based on the (a) statistical, (b) deep, (c) combined, and (d) selected set of features.

**Figure 8:** Receiver operating characteristic (ROC) curves based on (a) statistical, (b) deep, (c) combined, and (d) selected set of features.

**Table 1:** Class sample sizes of the dataset.

Class	Label	Dataset samples		After augmentation	
No disease/healthy	0, H	1227	26.26%	2454	34.53%
Bacterial pneumonia	1, B	2238	47.90%	2238	31.45%
Viral pneumonia	2, V	1207	25.84%	2414	33.97%

The article "A Pneumonia Diagnosis Scheme Based on Hybrid Features Extracted from Chest Radiographs Using an Ensemble Learning Algorithm" was published in 2021. Journal: J Healthc Eng.

**Table 2:** Classification outcomes based on different sets of features.

Feature set	Accuracy (%)	Precision (%)	Sensitivity (%)	Specificity (%)	F-score (%)
Statistical	82.13	82.16	81.94	93.03	82.05
Deep	83.02	80.56	82.83	93.38	82.92
Combined	86.30	86.15	85.91	95.60	86.03
Selected	85.79	85.61	85.40	95.36	85.51

**Table 3:** Parameters of the tuned RandomForest algorithm used for pneumonia classification.

Parameter	Value
n_estimators	200
Criterion	“Entropy”
max_features	“sqrt”
min_samples_split	2
min_samples_leaf	1
random_state	9
Verbose	0

**Table 4:** Classwise performance of the proposed method.

Class	Precision (%)	Sensitivity (%)	Specificity (%)	F-score (%)
H	88.34	96.74	93.27	92.35
B	84.97	72.32	94.11	78.14
V	85.15	88.67	92.05	86.87

**Table 5:** Performance comparison with other similar methods.

Reference	Identified classes	Number of samples	Classification model	Accuracy (%)	F-score (%)	Specificity (%)
[1]	N–P	5856	Multichannel CNN	97.92	97.97	—
[8]	N–P	5232	Inception V3	92.80	—	90.10
[8]	B–V	3883	Inception V3	90.70	—	90.90
[10]	N–P	5232	Ensemble of multiple CNNs	96.39	96.35	—
[11]	N–P	5857	Ensemble of convolutions with capsules	95.90	—	—
[12]	N–P	5856	PneumoniaNet	94.80	95.90	96.70
[13]	N–P	112, 120	MD-Conv	93.40	—	86.80
[13]	B–V	—	MD-Conv	91.00	—	92.60
[14]	N–P	5856	Custom CNN	93.73	—	—
[15]	H–B–V	6161	CovXNet	91.70	92.60	93.60
[15]	H–B–V	6161	ResidualNet	86.30	87.40	93.50
[15]	H–B–V	6161	InceptionNet	81.10	78.90	86.20
[15]	H–B–V	6161	VGG-19	79.80	77.90	83.40
[16]	H–B–V	5840	Model 1	85.26	89.00	—
[16]	H–B–V	5840	Model 2	92.31	94.00	—
[16]	H–B–V	5840	ResNet50	77.56	—	—
[16]	H–B–V	5840	Inception-v3	70.99	—	—
Proposed	H–B–V	4672	CNN + RandomForest	86.30	86.03	95.60

“--” denotes that the information is not mentioned in the associated study.

## Data Availability

The chest radiograph image dataset used to support the findings of this study is collected from a Kaggle repository entitled “Chest X-rays: bacterial/viral pneumonia/normal,” which was published in October 2020. K. Diamantaras, “Chest Xrays: bacterial/viral pneumonia/normal | Kaggle,” 2020. https://www.kaggle.com/kostasdiamantaras/chest-xrays-bacterial-viral-pneumonia-normal (accessed Dec. 29, 2020).
